# Cerebral blood flow alteration following acute myocardial infarction in mice

**DOI:** 10.1042/BSR20180382

**Published:** 2018-09-05

**Authors:** Abdullah Kaplan, Andriy Yabluchanskiy, Rana Ghali, Raffaele Altara, George W. Booz, Fouad A. Zouein

**Affiliations:** 1 Department of Pharmacology and Toxicology, American University of Beirut Faculty of Medicine, Beirut, Lebanon; 2 Translational Geroscience Laboratory, Reynold’s Oklahoma Center on Aging, Department of Geriatric Medicine, Oklahoma City, OK, U.S.A.; 3 Institute for Experimental Medical Research, Oslo University Hospital and University of Oslo, Oslo, Norway; 4 KG Jebsen Center for Cardiac Research, Oslo, Norway; 5 Department of Pathology, School of Medicine, University of Mississippi Medical Center, Jackson, MS, U.S.A.; 6 Department of Pharmacology and Toxicology, University of Mississippi Medical Center, School of Medicine, Jackson, MS, U.S.A.

**Keywords:** Aging, Cardiac Output, cerebral blood flow, myocardial infarction, right common coronary artery flow

## Abstract

Heart failure is associated with low cardiac output (CO) and low brain perfusion that imposes a significant risk for accelerated brain ageing and Alzheimer’s disease (AD) development. Although clinical heart failure can emerge several years following acute myocardial infarction (AMI), the impact of AMI on cerebral blood flow (CBF) at early stages and up to 30 days following MI is unknown. Sixteen months old male mice underwent left anterior descending (LAD) coronary artery ligation. Hemodynamics analyses were performed at baseline and at days 1, 7, and 30 post-MI. Left ventricular (LV) ejection fraction (EF), LV volumes, CO, and right common carotid artery (RCCA) diameter were recorded by echocardiography. RCCA flow (RCCA FL) was measured by Doppler echocardiography. LV volumes consistently increased (*P*<0.0012) and LV systolic function progressively deteriorated (*P*<0.0001) post-MI. CO and RCCA FL showed a moderate but significant decrease over the course of MI with similar fluctuation pattern such that both variables were decreased at day 1, increased at day 7, and decreased at 30 days post-MI. Correlation and regression analyses between CO and RCCA FL showed a strong correlation with significance at baseline and day 30 post-MI (*R* = 0.71, *P*=0.03, and *R* = 0.72, *P*=0.03, respectively). Days 1 and 7 analyses between CO and RCCA FL showed moderate correlation with non-significance post-MI (*R* = 0.51, *P*=0.2, and *R* = 0.56, *P*=0.12, respectively). In summary, CBF significantly decreased following AMI and remained significantly decreased for up to 30 days, suggesting a potential risk for brain damage that could contribute to cognitive dysfunction later in life.

## Introduction

Appropriate tissue blood perfusion is necessary for normal organ functions and is dependent on several factors including cardiac output (CO), blood volume, systemic blood pressure (BP), and local vasculature autoregulation, all of which positively depend on metabolic demand [1,2]. Distinct amongst other organs, the brain requires a constant supply of oxygen and nutrients due to its limited substrate storage capacity and high metabolic activity [3]. Despite the fact that the brain contributes only 2% to total body weight, it receives approximately 12% of the CO [4].

Cerebral perfusion is supplied by two carotid arteries and two vertebral arteries. Each carotid artery supplies approximately 40% to the total cerebral perfusion, while the two vertebral arteries supply the remaining 20% [5]. Cerebral blood flow (CBF) regulation is an integrative and multifaceted process that combines the function of multiple processes including pulmonary gas exchange, cardiovascular function, and intracranial cerebrovascular regulators [3]. Although CO and mean arterial pressure (MAP) are interrelated hemodynamic parameters that could exert simultaneous effects on CBF [4], multiple studies have revealed that the strongest correlation with CBF belonged to CO, especially in conditions with low CO such as heart failure disease [4,6,7]. In addition, several studies reported that therapies targetted at improvement of CO, including pharmacological interventions, cardiac transplantation, and cardiac resynchronization therapy, exerted a positive effect on improvement of CBF [8–10].

Recent studies suggest that impaired CBF as a result of CO reduction in heart failure patients may be a critical risk factor for Alzheimer’s disease (AD) development and accelerated brain ageing processes [11]. To date, no treatment is available to stop or reverse AD progression and consequently, preventive therapy is highly warranted [11,12]. Linking MI-induced CO reduction and subsequent CBF reduction to potential AD development and brain ageing in later stages of life is rational and worth investigating. Of note, cumulative heart failure rates of development 1 year following acute coronary syndrome hospitalization were 23.4% in ST-elevation myocardial infarction, 25.4% in non-ST-elevation myocardial infarction, and 16% in unstable angina patients in spite of interventional and pharmacological modern therapy [13]. Early diagnosis and accurate medical treatment of risk factors such as low CO levels can reduce the prevalence of AD and delay disease progression. In fact, it was projected that if intervention delays disease onset by 1 year, there would be 9 million fewer cases of AD by 2050 [11,12,14,15].

At the onset of MI, cardiac function, measured by CO and other hemodynamic parameters, rapidly deteriorates and persists until progressive restoration through medical intervention [13,16,17]. Depending on the infarct size and time to intervention, left ventricular (LV) remodeling post-MI is characterized by LV chamber size, shape, and function alterations subsequent to genomic, molecular, cellular, and interstitial changes [18,19]. In spite of full cardiac function restoration following acute medical intervention, clinical manifestation of heart failure development and its ramifications can progressively occur and be fully established in years following the onset of MI in patients [20]. Changes in the CBF as a result of CO deterioration with acute MI may have strong implications on the brain function; however, these changes have not been thoroughly investigated and remain poorly understood. Thus, it is critical to determine the CBF status in early stages of MI-induced CO reduction in order to prevent unnoticed early brain injury development that could translate to brain ageing and AD in later stages of life.

In addition to direct alteration of CO through myocardial mechanical injury and LV remodeling [19,21,22], MI induces a systemic inflammation and an elevated renin–angiotensin–aldosterone system (RAAS) activation affecting the remote organs including kidneys and the brain, and have been directly linked to brain perfusion impairment [4,23–26]. Although a strong correlation between chronic heart failure and CBF alteration has been established, no existing data link CO to CBF post-MI through the main phases of MI-induced cardiac remodeling including the inflammatory, granulation, and wound-healing phases [27]. This is the first study to serially investigate the hemodynamic impact of acute MI on CBF as early as day 1 and up to 30 days post-MI.

## Materials and methods

### Experimental animals

All animal experiments and procedures were performed according to an experimental protocol approved by AUB Institutional Animal Care and Use Committee in compliance with the Guide for Care and Use of Laboratory Animals of the Institute for Laboratory Animal Research of the National Academy of Sciences, U.S.A. Mice were allocated into two groups: study group (*n*=9) and sham operated group (*n*=6). Sixteen months old C57BL/6J male mice weighing 30–35 g underwent left anterior descending (LAD) coronary artery ligation surgery as previously described [28,29]. The age of experimental animals was chosen to represent translational power of our study and to mimic the average age of 50–55 years of MI incidence in humans [30]. Doppler echocardiography assessment was conducted at baseline, days 1, 7, and 30 post surgery. All animals were killed at day 30 post-MI after echocardiographic recording and BP measurements. Mouse model of MI is well-established and characterized by progressive increase in LV dilatation concomitantly with LV function deterioration similar to those observed in human patients [31]. Sham surgery was performed following the same procedure; however, the suture was passed underneath the LAD without ligation. Sham operated mice were killed 7 days post-op following echocardiographic recording and Doppler measurement.

### Blood pressure

Arterial BP was measured non-invasively using tail cuffs and volume pressure recording sensor technology and CODA high-throughput monitor, (Kent Scientific, Torrington, CT). Measurements were performed at day 30 post-MI in restrained and conscious experimental animals. Real-time measurements of systolic, diastolic, and MAP were recorded. Any irregular recording noted as false recording by the system were excluded.

### Echocardiography and Doppler echocardiography

Transthoracic echocardiography was performed using Vevo 2100™ High-Resolution Imaging System (Visual Sonics, Toronto, Canada). Mice were anesthetized with 1–2% isoflurane in an oxygen mix and placed on an electrical heated platform. B-mode (2D) images of left ventricle were acquired from the parasternal long axis view in supine position. Right common carotid artery (RCCA) was acquired from B-mode imaging in supine position (Figure 1A). Body temperature, heart rate, and respiratory rate were continuously monitored throughout the procedure via Indus MouseMonitor Heated Surgical Platform and the depth of anesthesia was adjusted accordingly. RCCA flow (RCCA FL) was recorded via Pulse-Wave Doppler (PWD) (Figure 1B). Color-wave Doppler was used to detect the direction of flow and PWD sample volume was aligned parallel to the direction of the flow using the angle-correction. Insonation angle was within the 60–70° range at baseline and at first day after surgery (D1), seventh day after surgery (D7), and thirtieth day after surgery (D30) post-MI. Peak velocity and velocity time integral (VTI) of flow in vessels were recorded for offline calculation. Three Doppler VTIs were measured and the mean of these measurements was used to calculate the RCCA FL. Two recorded carotid Doppler measurements at day 1 data were discarded due to low signal quality and artifacts.

**Figure 1:** Echocardiography and Doppler echocardiography image display (**A**) B-mode (2D) echocardiographic image of the RCCA. Arrow on the right side indicates the RCCA. (**B**) Doppler echocardiographic image of RCCA FL.

LV volumes were calculated based on modified ellipsoid (Teichholz) formula [32]:

$$LVEDV\;(\mu l)\;=\;7.0/\left(2.4\;+\;LVID;d\right)\;\times \;LVID;d^{3}$$

$$LVESV\;(\mu l)\;=\;7.0/(2.4\;+\;LVID;s)\;\times \;LVID;s^{3}$$

(LVID;d, LV internal diameter at the end diastolic phase; LVID;s, LV internal diameter at the end systolic phase).

LV stroke volume (SV) and ejection fraction (EF) were derived from the LV end diastolic volume (LVEDV) and LV end systolic volume (LVESV).

SV (μl) = LVEDV − LVESV

EF (%) = (SV/LVEDV) × 100

CO was derived from multiplication of SV and heart rate.

CO (ml/min) = SV × HR

where HR is heart rate.

RCCA was assumed to be a cylinder, and its cross-sectional area was calculated based on the following formula:

$$RCCA\;\;CSA\;=\;\pi \;\times \;R^{2}$$

[33], where CSA is cross-sectional area. R stands for the radius of artery that was obtained from the site of artery where the Doppler flow was recorded. CSA of RCCA was measured during three cardiac cycles and averaged.

RCCA FL was calculated based on the following equation:

RCCA  FL  (ml/min) = CSA × VTI × HR

[33,34], where CSA is cross-sectional area and HR is heart rate.

Fractional RCCA FL was calculated according to following equation:

Fractional  RCCA  FL (%) = (RCCA  FL/CO) × 100

### Infarct size measurement

Following the removal of the right ventricle, the left ventricle was sliced along its longitudinal axis and immersed for 5 min at 37°C in 2,3,5-triphenyl-2H-tetrazolium chloride (TTC) (5 mg/ml) for demarcation of infarcted region. The infarcted region was defined as the unstained section following incubation with TTC. ImageJ software (National Institutes of Health, Bethesda, MD) was used for infarct size measurement. The whole LV area along with the unstained region was traced and the measurement was done automatically by the program in pixels. The infarct area was expressed as a percentage of the left ventricle.

### Statistical analyses

When appropriate, correlation and regression analyses were performed. The correlation (R) and regression (R^2^) coefficients <0.3 were considered weak, >0.3 and <0.6 were considered moderate, and >0.6 were considered strong. The R^2^ and *P*-values in corresponding regression analysis represent goodness-of-fit and significance of the regression model. For multiple groups comparison, we used one-way ANOVA followed by Tukey’s post-hoc. Data are expressed as mean ± S.D. Analyses were done using GraphPad Prism version 7.03 for Windows (GraphPad Software, San Diego, CA, www.graphpad.com); a *P*-value of <0.05 was considered statistically significant in all analyses.

## Results

Data presented in this section are summarized in Tables 1 and 2. In agreement with other groups and confirming our previous data [28,29,31], we observed a progressive LV remodeling over the course of 30 days after initiation of MI. LV remodeling was evidenced by consistently increasing LV volumes (R = 0.99, R^2^ = 0.98, *P*<0.0012) and progressively deteriorating systolic function measured by EF (Figure 2, R = −0.73, R^2^ = 0.53, *P*<0.0001) and CO (Figure 3). Unlike study group, sham operated mice showed preserved LV systolic function during 7 days post-op (Figure 9).

**Figure 2:** Myocardial infarction resulted in a significant LV systolic dysfunction, which persistently deteriorated over the course of 30 days post-MI and was associated with increasing LVEDV

**Figure 3:** Both CO and RCCA FL fluctuated with the similar pattern through the time course of the MI

**Table 1:** Mean value of echocardiography and Doppler echocardiography before and after coronary artery ligation

Days	LVEDV (μl)	EF (%)	CO (ml/min)	RCCA VTI (mm)	RCCA FL (ml/min)	Fractional RCCA FL (%)
**BL**	73.3 ± 10.5	60.1 ± 8	17.7 ± 2.7	24.6 ± 5.6	1.9 ± 0.3	11.1 ± 1.4
**D1**	88.5 ± 10.6	33.3 ± 8.4	12.2 ± 2.5	17 ± 3	1.5 ± 0.3	12.1 ± 2.5
**D7**	107.8 ± 19.3	31.6 ± 9.2	13 ± 2.6	20.5 ± 2.4	1.6 ± 0.4	12.8 ± 2.6
**D30**	126 ± 34.9	26.9 ± 10.3	10.9 ± 2.9	19 ± 4.2	1.4 ± 0.4	13.2 ± 2.5

Abbreviation: BL, baseline data before surgery.

**Table 2:** Hemodynamic and tissue data from mice at day 30 after coronary artery ligation

Value	EF (%)	CO (ml/min)	RCCA VTI (mm)	RCCA FL (ml/min)	Fractional RCCA FL (%)	MAP (mmHg)	IS (%)
**Mean**	26.900401	10.876775	24.6192521	1.40587244	13.19309	99.89065256	31.87315
**S.D.**	10.258941	2.8690202	5.60544781	0.37940565	2.507708	12.18997185	10.47498
**Median**	31.44843	12.290591	22.125732	1.28584114	13.65738	95.75	32.03883
**Minimum**	13.110896	7.310145	18.140951	0.99289126	9.371708	87.71428571	20.73171
**25% quartile**	15.637963	7.6323335	21.485325	1.10119883	10.58362	90.84722222	21.52882
**75% quartile**	35.382087	13.59373	29.613539	1.74095098	14.78823	107.4285714	41.71212
**Maximum**	40.392202	14.04354	34.534877	2.06574576	16.98059	126.2	48.73418

Abbreviation: IS, LV infarct size.

We then investigated the impact of impaired LV systolic function on brain perfusion and measured the RCCA FL via Doppler echocardiography. Similar to CO, the RCCA FL showed a moderate but significant decrease over the course of MI with similar fluctuation pattern observed on days 1, 7, and 30 post-MI when compared with baseline (Figure 3, R = −0.61, R^2^ = 0.37, *P*<0.0001, R = −0.44, R^2^ = 0.19, *P*<0.0082, respectively). In sham operated mice however, both RCCA FL and CO fluctuated during 7 days post-op while remaining within the baseline level (Figure 9). We observed a strong positive correlation between CO and RCCA FL at baseline and at day 30 (R = 0.71 and R = 0.72, Figure 4A,D), and a moderate positive correlation at days 1 and 7 post-MI (R = 0.51 and R = 0.56, Figure 4B,C). However, in sham operated mice, a strong and positive correlation between CO and RCCA FL was observed at baseline, days 1 and 7 post-op (R = 0.82, R = 0.82, and R = 0.84, respectively. Figure 10A–C). While not significant, the fractional RCCA FL (%) showed a steady trend to increase from the baseline and to day 30 post-MI (Figure 5). The correlation between fractional RCCA FL (%) and CO was negative and moderate with no linear change (Figure 6, R = −0.44, R^2^ = 0.2, *P*=0.2).

**Figure 4:** Cumulative representation of correlations between RCCA FL and CO at baseline, days 1, 7, and 30 post-MI (**A**) RCCA FL positively and significantly correlated with CO at baseline. (**B**,**C**) RCCA FL moderately and positively but not significantly correlated with CO at days 1 and 7 post-MI. (**D**) RCCA FL positively and significantly correlated with CO at day 30 post-MI.

**Figure 5:** Fractional RCCA FL steadily and mildly increased over the course of 30 days post-MI There were no significant differences between days post-MI when compared with baseline.

**Figure 6:** The correlation between fractional RCCA FL (%) and CO was negative, moderate, and non-significant with no linear change

Both CO and RCCA FL were inversely correlated with the infarct size (R = −0.81, R^2^ = 0.65, *P*=0.0091, R = −0.57, R^2^ = 0.33, *P*=0.10, respectively). However, the relationship of these changes was only significant for the CO (Figure 7A,B). Finally, MAP and flow in the right coronary artery assessment at day 30 post-MI revealed no correlation (Figure 8, R = −0.31, R^2^ = 0.10, *P*=0.40).

**Figure 7:** Representation of the correlation between CO and infarct size, and between RCCA FL and infarct size, 30 days post-MI (**A**) CO negatively and significantly correlated with the infarct size at day 30 post-MI. (**B**) RCCA FL negatively, but non-significantly correlated with the infarct size at day 30 post-MI.

**Figure 8:** RCCA FL did not correlate with MAP at day 30 post-MI

## Discussion

Following MI in all mammals, ischemic hearts undergo an intensive structural and functional remodeling in three major phases: inflammatory phase (1–3 days); granulation phase (1–7 days); and maturation/wound healing phase (weeks) [24,27]. Although LV remodeling starts at the onset of MI, clinical manifestation of chronic heart failure may not develop for years in humans given the progressive maladaptive remodeling that may continue for a lifetime [20]. Multiple studies revealed the association between CO and CBF in both healthy and cardiac impaired individuals linking heart failure mediated low CO to CBF reduction [4,6–10]. However, no studies assessed the impact of early (day 1) till late stages (30 days) of acute cardiac injury post MI, on CBF. The findings reported in this manuscript are novel, showing for the first time the CBF through RCCA as early as day 1 and up to 30 days post-MI.

The major finding of the present study is that CBF decreases at the onset of MI and remains lower than baseline for 30 days (Table 1/Figure 3). Our findings correlate well with others who reported reduction in CBF 4–6 weeks after MI and before any signs of congestive heart failure development [35]. Interestingly, although SV, CO, and RCCA FL significantly decreased at day 1 post-MI and remained lower than baseline for 30 days, fractional RCCA FL (%) mildly but steadily and non-significantly increased, reaching its highest level at day 30 post-MI (Table 1/Figure 5). This means that the percentage of blood derived to the brain from total circulating blood increased after MI, but the amount of blood perfusing the brain decreased in-line with cardiac dysfunction. These findings indicate that CBF is directly associated with cardiac remodeling, functional stages, and the associated systemic compensatory mechanisms following MI. However, CBF regulatory mechanisms were not able to restore complete cerebral blood supply under low cardiac function and known inflammatory conditions accompanying MI since CBF remained lower than the baseline 30 days following MI (Table 1). Unlike previous reports where CO and fractional CBF inversely and significantly correlated with healthy individuals, our data showed no significant correlation between these parameters suggestive of unknown MI-related systemic regulation blunting mechanisms (Figure 6) [36].

Systemic regulatory mechanisms following both cardiac dysfunction and decrease in major organ blood perfusion are well documented [37,38]. Decrease in SV at the onset of MI triggers immediate autonomic activity characterized by catecholamine discharge and subsequent increase in heart rate and vasoconstriction [25]. Persistent hypoperfusion elicits a long-term compensatory mechanism involving the RAAS that promotes vasoconstriction, renal salt and water retention, and overall increase in blood volume [25,39,40]. Within the context of MI, compensatory mechanisms can either fully or partially restore CO depending on the infarct size and the absence or presence of comorbidities [24]. In-line with previous reports, our findings showed a strong correlation between CO and CBF, 4 weeks post-MI [24,35] (Figure 4). The effects of regulatory mechanisms were noticed in our hemodynamic analyses. For instance, in comparison with day 1 post-MI, we observed improved CO and RCCA FL at day 7 of cardiac remodeling notwithstanding increased LV dilatation (Figure 3). Interestingly, unlike the correlation at BL and day 30 post-MI, the correlation between CO and RCCA FL at days 1 and 7 post-MI was moderate and not statistically significant (opposite to what was observed in sham operated mice) (Figures 4 and 9). These data suggest that in the first and second stages of cardiac remodeling post-MI, regulatory mechanisms limit the impact of CO on CBF. In fact, CBF is an integrative and complex process combining the function of multiple systems including pulmonary gas exchange, cardiovascular function, and intracranial cerebrovascular regulators [3,4]. MI impact on cerebral perfusion is multifaceted and not only mediated through CO alteration. Individuals with MI experience a high level of cardiac and systemic inflammation that alters CBF in spite of the acute and long-term compensatory mechanisms that improve cerebral vascular beds perfusion [4,21,23,25]. Unlike early stages of MI that involve a vicious systemic inflammatory response including circulating pro-inflammatory cytokines, chemokines, and cell adhesion molecules, as well as peripheral leukocytes and platelets activation [21], later phases of cardiac remodeling post-MI are more settled with different inflammatory and functional properties. The multi-remodeling phases could explain the variation in CO and RCCA FL correlation in different stages post-MI [19,21,22]. In-line with infarct size impact, unlike the strong inverse and significant correlation with CO, a weak, inverse, and non-significant correlation was noticed with RCCA FL at day 30 post-MI (Figure 7). These findings suggest that infarct size is a good predictor of CO but not of CBF. Correlation between infarct size and RCCA FL is most probably weakened by MI-mediated multiple effects such as LV remodeling and its impact on regulators of cerebral perfusion.

**Figure 9:** Both CO and RCCA FL fluctuated within baseline levels through the time course of the wound healing post-sham operation

With respect to BP variation and its impact on CBF, patients with uncomplicated MI and intact autonomic nervous system are usually normotensive [39]. Our findings were similar to what has been previously reported [35] with normal BP at 30 days post-MI and hence no correlation between CBF and MAP was noticed (Figure 8).

In summary, intact compensatory and regulatory mechanisms were not able to restore normal CBF in mouse model of 30 days of MI. These findings emphasize the importance of an appropriate intervention at cerebral, cardiac, and/or systemic level including inflammatory resolution to immediately restore CBF post-MI and prevent cerebral hypoperfusion ramifications on potential acute or time-dependent cerebral injury.

### Strengths and weaknesses of the study

Although several imaging techniques are currently available to assess CBF [41], Doppler ultrasound is a non-invasive, accurate, and very reliable method to assess CBF [42]. Blood flow volume in the internal carotid artery is an indicator of CBF in the corresponding hemisphere as shown in linear correlation with ^133^Xe clearance technique [42,43]. Common carotid artery is divided into internal and external carotid arteries. While internal carotid artery supplies blood to the majority of the cerebral cortex, external carotid artery supplies blood to the face, scalp, scull, and meninges. These two vascular beds appear to have different regulatory mechanisms in controlling blood flow [44–46]. Previous reports suggest that external cerebral vasculature plays a dynamic role in intracranial CBF regulation [44,47]. In fact, it was shown that changes in external carotid artery are more distinctive than internal carotid artery changes under acute hypotensive and hypertensive conditions in healthy individuals [44,47]. However, external carotid artery regulation against BP fluctuation may not be enough to restore the internal carotid artery flow under chronic condition such as heart failure where CO and not BP alteration prevail.

In the present study, common carotid artery but not internal carotid artery was used for flow measurement given the easier access due to the size of the animal studied and as previously reported [34,42]. Interestingly, CBF does not reduce uniformly in patients with heart failure with the right hemisphere being more affected [48]. Multiple studies reported that heart failure induces more damage on the right side of brain affecting structures responsible for autonomic nerve regulation [48,49]. Therefore the RCCA was used for CBF assessment in our study. Although, BP measurement was conducted only at the end of the present study to limit stress impact, the findings might be confounded by potential simultaneous change in BP during the time course of the study. However, it is worth noting that, previous studies showed a better correlation between CO and CBF than between arterial BP and CBF [4]. Additionally, augmentation of a low CO showed a stronger impact on CBF than did the increase in arterial BP [4]. Another important factor that was not within the scope of this study was systemic inflammation associated with MI. Systemic inflammation is known to be a major player in cerebral perfusion alteration and the increase in cerebrovascular resistance [6,21,50,51]. Systemic inflammatory and its impact on cerebrovascular perfusion at multiple time points post-MI was not the goal of this study and therefore was not assessed.

With regard to anesthesia, CO and RCCA FL were measured under isoflurane inhalation. Isoflurane is known to reduce systemic vascular resistance and produce minimal cardiac depression [52,53]. Although experiments were conducted under identical conditions, a possible impact of isoflurane on the relationship between CO and RCCA FL cannot be ruled out.

With respect to CO and CBF relationship, previous report showed that CO and CBF relationship was different at rest and during exercise in healthy individuals [54]. The authors documented that the changes in vascular resistance was greater in the brain than in the forearm at the same perfusion pressure during exercise. In other words, authors believe that CO fluctuation minimally affect CBF during exercise simply because of the small proportion of total CO being directed to the brain. However, in disease state, a clinical study showed that physical exercise may impair cerebral perfusion in patients with chronic heart failure because of their reduced ability to increase CO [55]. Further investigation to disclose the impact of exercise on cerebral perfusion shortly after MI and before heart failure establishment is warranted especially when physical exercise is currently considered a standard rehabilitation program post-MI [56,57].

Although CO and CBF are directly connected, one cannot rule out the effect of aortic compliance on the heart–CBF transition. Under physiological conditions, the blood volume is ejected from the left ventricle into the central arteries such as aorta and carotid arteries and transmitted to the brain with minimal pulsatile fluctuation. In fact, attenuated hemodynamics fluctuation at the cerebrovascular level is an important determinant of cerebrovascular health [58–61]. Tomoto et al. [61] showed that endurance exercise prevents brain perfusion pulsatile stress due to greater aortic compliance. The arterial compliance/dispensability is influenced by the sympathetic nervous impact on the smooth muscle tone [60]. Sugawara et al. [60] showed that systemic vasoconstriction induced by applying lower body negative pressure deteriorates the dampening effect on cerebral pulsatile hemodynamics in healthy individuals. Therefore, the enhanced sympathetic activation normally observed post-MI may have an impact on dampening effect of aorta and carotid arteries that may transmit high pulsatile stress to brain. However, compromised LV pumping function post-MI leads to reduced SV which is anticipated to offset the impact of augmented aortic stiffness due to enhanced sympathetic activation.

Last but not the least, in order to eliminate the impact of surgical stress on the relationship between CO and RCCA FL, a sham group was included in the present study. Both CO and RCCA FL fluctuated within the baseline levels till day 7 post-op (Figure 9). We also observed a strong and significant correlation between CO and RCCA FL at baseline and the days post-op (Figure 10). These findings confirm the fact that the non-significant correlation observed at day 1 and 7 post MI between CO and RCCA FL was due to MI and/or the conditions accompanying MI.

**Figure 10:** Cumulative representation of correlations between RCCA FL and CO at baseline, days 1 and 7 post-sham operation (**A**) RCCA FL positively and significantly correlated with CO at baseline, (**B**) at day 1, and (**C**) at day 7 post-sham operation.

## Conclusion and future direction

Our novel findings report the association between CBF and CO in early stages of cardiac remodeling and up to 30 days following acute MI. We showed that CBF significantly decreased along with CO following acute MI; however, regulatory systems could not restore CBF completely following reduced CO. The present study highlights the importance of impaired CBF at early and advanced stages of acute MI and its potential impact on cerebrovascular prognosis. Early intervention to fully restore normal CBF following acute MI is critical and warrant future investigation.

## Abbreviations

AD: Alzheimer’s disease
BP: blood pressure
CBF: cerebral blood flow
CO: cardiac output
EF: ejection fraction
LAD: left anterior descending
LV: left ventricular
MAP: mean arterial pressure
PWD: pulse-wave Doppler
RAAS: renin–angiotensin–aldosterone system
RCCA: right common carotid artery
RCCA FL: RCCA flow
SV: stroke volume
TTC: 2,3,5-triphenyl-2H-tetrazolium chloride
VTI: velocity time integral

## References

[1] Bryan-BrownC.W. (1988) Blood flow to organs: parameters for function and survival in critical illness. Crit. Care Med. 16, 170–178 10.1097/00003246-198802000-00016 3277775

[2] MathiasC.J. (2000) Cerebral hypoperfusion and impaired cerebral function in cardiac failure. Eur. Heart J. 21, 346 10.1053/euhj.1999.1960 10666345

[3] WillieC.K. (2014) Integrative regulation of human brain blood flow. J. Physiol. 592, 841–859 10.1113/jphysiol.2013.268953 24396059PMC3948549

[4] MengL. (2015) Cardiac output and cerebral blood flow: the integrated regulation of brain perfusion in adult humans. Anesthesiology 123, 1198–1208 10.1097/ALN.0000000000000872 26402848

[5] ZaunerA. and MuizelaarJ.P. (1997) Brain metabolism and cerebral blood flow. In Head Injury (ReillyP. and BullockR., eds), Chapman & Hall, London

[6] ChoiB.R. (2006) Factors associated with decreased cerebral blood flow in congestive heart failure secondary to idiopathic dilated cardiomyopathy. Am. J. Cardiol. 97, 1365–1369 10.1016/j.amjcard.2005.11.059 16635612

[7] LoncarG. (2011) Relationship of reduced cerebral blood flow and heart failure severity in elderly males. Aging Male 14, 59–65 10.3109/13685538.2010.511326 20873985

[8] GruhnN. (2001) Cerebral blood flow in patients with chronic heart failure before and after heart transplantation. Stroke 32, 2530–2533 10.1161/hs1101.098360 11692012

[9] van BommelR.J. (2010) Effect of cardiac resynchronization therapy on cerebral blood flow. Am. J. Cardiol. 106, 73–77 10.1016/j.amjcard.2010.02.015 20609651

[10] ZuccalaG. (2005) Use of angiotensin-converting enzyme inhibitors and variations in cognitive performance among patients with heart failure. Eur. Heart J. 26, 226–233 10.1093/eurheartj/ehi058 15618043

[11] JeffersonA.L. (2010) Cardiac output as a potential risk factor for abnormal brain aging. J. Alzheimers Dis. 20, 813–821 10.3233/JAD-2010-100081 20413856PMC3041147

[12] QiuC. (2006) Heart failure and risk of dementia and Alzheimer disease: a population-based cohort study. Arch. Intern. Med. 166, 1003–1008 10.1001/archinte.166.9.1003 16682574

[13] KaulP. (2013) Incidence of heart failure and mortality after acute coronary syndromes. Am. Heart J. 165, 379–385.e2 10.1016/j.ahj.2012.12.00523453107

[14] BrookmeyerR. (2007) Forecasting the global burden of Alzheimer’s disease. Alzheimers Dement. 3, 186–191 10.1016/j.jalz.2007.04.381 19595937

[15] CermakovaP. (2015) Heart failure and Alzheimer’s disease. J. Intern. Med. 277, 406–425 10.1111/joim.12287 25041352PMC4409079

[16] CahillT.J. and KharbandaR.K. (2017) Heart failure after myocardial infarction in the era of primary percutaneous coronary intervention: mechanisms, incidence and identification of patients at risk. World J. Cardiol. 9, 407–415 10.4330/wjc.v9.i5.407 28603587PMC5442408

[17] GerberY. (2013) Contemporary trends in heart failure with reduced and preserved ejection fraction after myocardial infarction: a community study. Am. J. Epidemiol. 178, 1272–1280 10.1093/aje/kwt109 23997209PMC3792728

[18] CohnJ.N., FerrariR. and SharpeN. (2000) Cardiac remodeling–concepts and clinical implications: a consensus paper from an international forum on cardiac remodeling. Behalf of an International Forum on Cardiac Remodeling. J. Am. Coll. Cardiol. 35, 569–582 10.1016/S0735-1097(99)00630-0 10716457

[19] FrangogiannisN.G. (2015) Pathophysiology of Myocardial Infarction. Compr. Physiol. 5, 1841–1875 10.1002/cphy.c150006 26426469

[20] GajarsaJ.J. and KlonerR.A. (2011) Left ventricular remodeling in the post-infarction heart: a review of cellular, molecular mechanisms, and therapeutic modalities. Heart Fail. Rev. 16, 13–21 10.1007/s10741-010-9181-7 20623185

[21] FangL. (2015) Systemic inflammatory response following acute myocardial infarction. J. Geriatr. Cardiol. 12, 305–312 2608985610.11909/j.issn.1671-5411.2015.03.020PMC4460175

[22] LiA.H. (2014) Dynamic changes in myocardial matrix and relevance to disease: translational perspectives. Circ. Res. 114, 916–927 10.1161/CIRCRESAHA.114.302819 24577970

[23] MurrayK.N. (2014) Systemic inflammation impairs tissue reperfusion through endothelin-dependent mechanisms in cerebral ischemia. Stroke 45, 3412–3419 10.1161/STROKEAHA.114.006613 25228257PMC4363555

[24] RichardsonW.J. (2015) Physiological implications of myocardial scar structure. Compr. Physiol. 5, 1877–1909 10.1002/cphy.c140067 26426470PMC4727398

[25] JacksonG. (2000) ABC of heart failure. Pathophysiology. BMJ 320, 167–170 10.1136/bmj.320.7228.167 10634740PMC1128747

[26] RupareliaN. (2013) Myocardial infarction causes inflammation and leukocyte recruitment at remote sites in the myocardium and in the renal glomerulus. Inflamm. Res. 62, 515–525 10.1007/s00011-013-0605-4 23471223PMC3625409

[27] AltaraR. (2016) Temporal cardiac remodeling post-myocardial infarction: dynamics and prognostic implications in personalized medicine. Heart Fail. Rev., 21, 25–47, 10.1007/s10741-015-9513-8 26498937

[28] KobeissyF. (2017) Acute exposure to cigarette smoking followed by myocardial infarction aggravates renal damage in an *in vivo* mouse model. Oxid. Med. Cell Longev. 2017, 5135241 10.1155/2017/5135241 29177025PMC5671747

[29] LindseyM.L. (2015) A novel collagen matricryptin reduces left ventricular dilation post-myocardial infarction by promoting scar formation and angiogenesis. J. Am. Coll. Cardiol. 66, 1364–1374 10.1016/j.jacc.2015.07.035 26383724PMC4575409

[30] DuttaS. and SenguptaP. (2016) Men and mice: relating their ages. Life Sci. 152, 244–248 10.1016/j.lfs.2015.10.025 26596563

[31] GaoX.M. (2000) Serial echocardiographic assessment of left ventricular dimensions and function after myocardial infarction in mice. Cardiovasc. Res. 45, 330–338 10.1016/S0008-6363(99)00274-6 10728353

[32] FollandE.D. (1979) Assessment of left ventricular ejection fraction and volumes by real-time, two-dimensional echocardiography. A comparison of cineangiographic and radionuclide techniques. Circulation 60, 760–766 10.1161/01.CIR.60.4.760 476879

[33] SoustielJ.F. (2002) A new angle-independent Doppler ultrasonic device for assessment of blood flow volume in the extracranial internal carotid artery. J. Ultrasound Med. 21, 1405–1412 10.7863/jum.2002.21.12.1405 12494983

[34] EickeB.M. (2001) Lack of association between carotid artery volume blood flow and cardiac output. J. Ultrasound Med. 20, 1293–1298, 10.7863/jum.2001.20.12.1293 11762541

[35] YangJ. (2012) Proximal cerebral arteries develop myogenic responsiveness in heart failure via tumor necrosis factor-alpha-dependent activation of sphingosine-1-phosphate signaling. Circulation 126, 196–206 10.1161/CIRCULATIONAHA.111.039644 22668972

[36] HenriksenO.M. (2014) Relationship between cardiac function and resting cerebral blood flow: MRI measurements in healthy elderly subjects. Clin. Physiol. Funct. Imaging 34, 471–477 10.1111/cpf.12119 24314236

[37] MentzR.J. and O’ConnorC.M. (2016) Pathophysiology and clinical evaluation of acute heart failure. Nat. Rev. Cardiol. 13, 28–35 10.1038/nrcardio.2015.134 26370473

[38] KopelT.H and OrganL.M. (2008) Perfusion in Acute Heart Failure Syndromes (Mebazaa AG.M., ZannadF.M. and ParrilloJ.E., eds), Springer, London

[39] YapY.G. (2007) Prognostic value of blood pressure measured during hospitalization after acute myocardial infarction: an insight from survival trials. J. Hypertens. 25, 307–313 10.1097/HJH.0b013e3280115bae 17211237

[40] E.M.A. and B.E., (1997). Acute myocardial infarction. In A Textbook of Cardiovascular Medicine, (B.E., ed) W.B. Saunders, Philadelphia

[41] WintermarkM. (2005) Comparative overview of brain perfusion imaging techniques. Stroke 36, e83–e99 10.1161/01.STR.0000177884.72657.8b 16100027

[42] WestraS.J. (1997) Carotid artery volume flow: *in vivo* measurement with time-domain-processing US. Radiology 202, 725–729 10.1148/radiology.202.3.9051025 9051025

[43] SoustielJ.F. (2003) Assessment of cerebral blood flow by means of blood-flow-volume measurement in the internal carotid artery: comparative study with a 133xenon clearance technique. Stroke 34, 1876–1880 10.1161/01.STR.0000080942.32331.39 12843349

[44] OgohS. (2014) Regional redistribution of blood flow in the external and internal carotid arteries during acute hypotension. Am. J. Physiol. Regul. Integr. Comp. Physiol. 306, R747–R751 10.1152/ajpregu.00535.2013 24598464

[45] OgohS. (2014) Hyperthermia modulates regional differences in cerebral blood flow to changes in CO_2_. J. Appl. Physiol. (1985) 117, 46–52 10.1152/japplphysiol.01078.2013 24790021

[46] SatoK. (2012) Differential blood flow responses to CO(2) in human internal and external carotid and vertebral arteries. J. Physiol. 590, 3277–3290 10.1113/jphysiol.2012.230425 22526884PMC3459042

[47] OgohS. (2017) Effect of increases in cardiac contractility on cerebral blood flow in humans. Am. J. Physiol. Heart Circ. Physiol. 313, H1155–H1161 10.1152/ajpheart.00287.2017 28916637PMC5814648

[48] SerberS.L. (2014) Cerebral blood flow velocity and vasomotor reactivity during autonomic challenges in heart failure. Nurs. Res. 63, 194–202 10.1097/NNR.0000000000000027 24785247PMC4024060

[49] WooM.A. (2003) Regional brain gray matter loss in heart failure. J. Appl. Physiol. (1985) 95, 677–684 10.1152/japplphysiol.00101.2003 12716866

[50] VogelsR.L. (2008) Transcranial Doppler blood flow assessment in patients with mild heart failure: correlates with neuroimaging and cognitive performance. Congest. Heart Fail. 14, 61–65 10.1111/j.1751-7133.2008.07365.x 18401213

[51] YndestadA. (2006) Systemic inflammation in heart failure–the whys and wherefores. Heart Fail. Rev. 11, 83–92 10.1007/s10741-006-9196-2 16819581

[52] IltisI. (2005) *In vivo* assessment of myocardial blood flow in rat heart using magnetic resonance imaging: effect of anesthesia. J. Magn. Reson. Imaging 22, 242–247 10.1002/jmri.20352 16028244

[53] RothD.M. (2002) Impact of anesthesia on cardiac function during echocardiography in mice. Am. J. Physiol. Heart Circ. Physiol. 282, H2134–H2140 10.1152/ajpheart.00845.2001 12003821

[54] OgohS. (2005) The effect of changes in cardiac output on middle cerebral artery mean blood velocity at rest and during exercise. J. Physiol. 569, 697–704 10.1113/jphysiol.2005.095836 16210355PMC1464249

[55] G.H. (1996) Physical exercise may impair cerebral perfusion in patients with chronic heart-failure. In Cardiology in the Elderly, vol. 4, Sweden

[56] AbelaM. (2018) Exercise training in heart failure. Postgrad. Med. J. 94, 392–397 10.1136/postgradmedj-2018-135638 29728451

[57] DagnerV., ClaussonE.K. and JakobssonL. (2018) Prescribed physical activity maintenance following exercise based cardiac rehabilitation: factors predicting low physical activity. Eur. J. Cardiovasc. Nurs. 10.1177/1474515118783936 29905494

[58] MitchellG.F. (2008) Effects of central arterial aging on the structure and function of the peripheral vasculature: implications for end-organ damage. J. Appl. Physiol. (1985) 105, 1652–1660 10.1152/japplphysiol.90549.2008 18772322PMC2584844

[59] O’RourkeM.F. and SafarM.E. (2005) Relationship between aortic stiffening and microvascular disease in brain and kidney: cause and logic of therapy. Hypertension 46, 200–204 10.1161/01.HYP.0000168052.00426.65 15911742

[60] SugawaraJ. (2017) Impact of mild orthostatic stress on aortic-cerebral hemodynamic transmission: insight from the frequency domain. Am. J. Physiol. Heart Circ. Physiol. 312, H1076–H1084 10.1152/ajpheart.00802.2016 28258058

[61] TomotoT. (2018) Relationship between aortic compliance and impact of cerebral blood flow fluctuation to dynamic orthostatic challenge in endurance athletes. Front. Physiol. 9, 25 10.3389/fphys.2018.00025 29422868PMC5788908

